# Mechanisms of Banxia Xiexin Decoction Underlying Chronic Atrophic Gastritis via Network Pharmacology, Molecular Docking, and Molecular Dynamics Simulations

This article has been retracted.

**DOI:** 10.1155/2022/4237040

**Published:** 2022-09-15

**Authors:** Cheng Chang, Weiqi Feng, Min Sun, Xiaowen Yu, Zhiguang Sun

**Affiliations:** ^1^Nanjing University of Chinese Medicine, Nanjing 210023, China; ^2^Jiangsu Provincial Second Chinese Medicine Hospital, The Second Affiliated Hospital of Nanjing University of Chinese Medicine, Nanjing 210017, China; ^3^Department of Respiration, Zhenjiang Hospital of Chinese Traditional and Western Medicine, Zhenjiang 212000, China; ^4^College of Special Education, Nanjing Normal University of Special Education, Nanjing 210038, China; ^5^Zhenjiang Hospital Affiliated to Nanjing University of Chinese Medicine, Zhenjiang 212000, China

## Abstract

Chronic atrophic gastritis (CAG) is a common chronically digestive disease which is notoriously characterized by atrophy of the epithelium and glands of the gastric mucosa, reduced number, thinning of the gastric mucosa, thickening of the mucosal base, or pyloric glandular hyperplasia and intestinal glandular hyperplasia, or with atypical hyperplasia. Banxia Xiexin decoction (BXD) has been applied for two thousand years and is considered an effective therapy for functional dyspepsia, gastroesophageal reflux disease and colon cancer. In this current study, to probe into the underlying mechanism of BXD on CAG, network pharmacology was conducted to collect druggable ingredients and predicted targets of BXD and the CAG-associated targets were harvested to take intersection with druggable ingredients from BXD predicted targets to obtain potential critical action targets. Subsequently, GO enrichment analysis and Kyoto Encyclopedia of Genes and Genomes pathway enrichment analysis were conducted to elucidate the underlying mechanisms and roles from the perspective of overall pathways and cellular functions. Eventually, molecular docking integrated with molecular dynamics simulations was conducted to further investigate the mechanism of action of BXD active ingredients on CAG from drug molecule-target interactions and to provide a theoretical basis for BXD drug development.

## 1. Introduction

Chronic atrophic gastritis (CAG) is a common chronically digestive disease which is notoriously characterized by atrophy of the epithelium and glands of the gastric mucosa, reduced number, thinning of the gastric mucosa, thickening of the mucosal base, or pyloric glandular hyperplasia and intestinal glandular hyperplasia, or with atypical hyperplasia [1, 2]. The representative clinical manifestation involved vague pain in the upper abdomen, fullness, belching, loss of appetite, wasting, anaemia, etc. [3]. It is a nonspecific and multicausal disease or precancerous lesion. Clinical and epidemiological evidence has suggested the repeated inflammation of gastric mucosa, Helicobacter pylori's infection, and gastric mucosal lesion induced by alcohol or an unhealthy diet are the dominating pathological factors of CAG [4, 5]. However, compared with the imperious command for the effective therapeutic approaches currently, there is still a lack of effective clinical therapy for CAG.

Traditional Chinese medicine (TCM) has been prevalently acknowledged as the treasure trove of natural compounds with pronounced clinical efficacy [6]. As reported before, many TCMs can improve CAG, such as berberine [7] and Jianpiyiqi formula [8]. Banxia Xiexin decoction (BXD), as a classic prescription Treatise on Febrile Diseases (Shanghan Lun), has been applied for two thousand years and is considered an effective therapy for functional dyspepsia, gastroesophageal reflux disease, and colon cancer [9–11]. Moreover, BXD has been documented to affect drug sensitivity in gastric cancer cells [12]. The classic TCM prescription BXD is composed of seven medicinal herbs, including *Pinelliae Rhizoma* (Ban Xia), *Coptidis Rhizoma* (Huang Lian), *Scutellariae Radix* (Huang Qin), *Zingiberis Rhizoma* (Gan Jiang), *Ginseng Radix* (Ren Shen), *Jujubae Fructus* (Da Zao), and *Glycyrrhizae Radix* (Gan Cao). Drawing on previous studies, BXD has yielded various anti-inflammatory and antioxidative pharmacological effects, and the therapeutic effects on CAG and Ulcerative colitis (UC) are confirmed evidence [11, 13]. Pharmacological research demonstrated that the master ingredient of BXD which encompasses alkaloids and flavonoids could exert therapeutic effects on CAG by regulating inflammatory response and protecting from H. pylori infection and interfering with H. pylori growth and virulence [14]. Nevertheless, the detailed mechanism of BXD on CAG remains unveiled.

Network pharmacology is an emerging method to shed light on the process of disease development from the perspective of scientific biology and the equilibrium of biological network, to understand drug-organism interactions from a holistic viewpoint of promoting or restoring the equilibrium of biological network, and to guide the discovery of new drugs, which coincides with the theory of Traditional Chinese Medicine and is widely utilized for the exploration of mechanisms of Traditional Chinese Medicine [15, 16]. Currently, with the prevalence and development of computational chemistry methods and the proposed theoretical basis of the computer-aided drug designing (CADD) receptor-ligand interaction hypothesis and molecular simulations, structural biology combined with kinetic simulation methods promotes the processes of drug discovery and elucidation of target interactions [17].

In our current study, network pharmacology was initially conducted to screen out potential druggable ingredients of BXD and probe into the underlying biological mechanism by which BXD on the treatment of CAG from a systemic perspective and at the molecular level. Subsequently, the herb-biological function network of BXD was established to illustrate the regulatory effect of BXD for the treatment of CAG. Key targets were selected to perform the molecular docking procedure for predicting binding energy and screening potential therapeutic ingredients. Eventually, the target-compound complexes were conducted molecular dynamics simulation and performed binding free energy calculations via Gromacs 2020 software and MMPBSA procedure.

## 2. Materials and Methods

### 2.1. Network Pharmacology Analysis

#### 2.1.1. Identification of the Active Compounds of BXD and Compound Data Collection

Bioinformatics was conducted to identify and comprehensively collect underlying therapeutic druggable compounds of BXD. The whole procedure was described as follows. Initially, the online database Traditional Chinese Medicine Systems Pharmacology Analysis Database and Analysis Platform (http://tcmspw.com/tcmsp.php) was conducted to screen potential active compounds from BXD by, respectively, importing *Pinelliae Rhizoma* (Ban Xia), *Coptidis Rhizoma* (Huang Lian), *Scutellariae Radix* (Huang Qin), *Zingiberis Rhizoma* (Gan Jiang), *Ginseng Radix* (Ren Shen), *Jujubae Fructus* (Da Zao), and *Glycyrrhizae Radix* (Gan Cao) as keywords [18]. Additionally, a literature search in PubMed Central of the NCBI database (https://www.ncbi.nlm.nih.gov/) was conducted as supplementary compounds of BXD. Eventually, all obtained compounds with the predicted drug properties were uploaded on ProTox-II (https://tox-new.charite.de/protox_II/index.php?site=home) which is an online database for predicting the toxicity of compounds [19]. Active compounds with low toxic doses and filtered with the criterion of oral bioavailability (OB ≥ 30%) and drug-likeness (DL ≥ 0.18) and the mol2 format files of selected active compounds were downloaded for further target prediction. Subsequently, macromolecular targets of active ingredients were predicted via SwissTargetPrediction (http://www.swisstargetprediction.ch/index.php) and PharmMapper Server (http://www.lilab-ecust.cn/pharmmapper/) which were prevalently utilized for potential target identification [20, 21]. Eventually, all prediction targets corresponding to components obtained from the above database search were imported into Venny 2.1 (https://bioinfogp.cnb.csic.es/tools/venny/index.html) to combine duplicate item.

### 2.2. CAG-Associated Target Collection

To comprehensively collect CAG-associated targets, six resources of disease online databases including CTD (http://ctdbase.org/), OMIM (http://omim.org/) DisGeNET (http://www.disgenet.org/), NCBI Gene (https://www.ncbi.nlm.nih.gov), and GENECARD (https://www.genecards.org/) were utilized by importing the keyword of chronic atrophic gastritis [22–24]. Considering that CAG is a type of chronic gastritis which exerts similar aetiology and pathology, we supplemented chronic gastritis-related targets and the overall aggregated targets were imported into Excel software for merging and removing repeated targets. The predicted potential targets for drugs of BXD and CAG-associated targets were derived from the intersection as potential targets of BXD on CAG.

### 2.3. Enrichment Analysis and Network Construction

Gene Ontology (GO) and Kyoto Encyclopedia of Genes and Genomes (KEGG) pathway enrichment analyses were conducted on the Metascape database (http://metascape.org) by importing key targets which refer to the intersection of CAG-related targets and BXD predicted targets [25]. GO- (Gene Ontology-) related biological processes (BP), cellular components (CC), molecular functions (MF) and KEGG pathways, GO enrichment, and KEGG pathway enrichment analyses were conducted to probe into the underlying mechanism of BXD in CAG at holistic systematic perspective, offering molecular mechanism demonstration for BXD treatment of CAG. To visualize the analysis results, RStudio was utilized for presenting enrichment analysis results. Eventually, the network that encompasses the association between active ingredients and corresponded targets was constructed via Cytoscape 3.7.1 software (http://www.cytoscape.org/) [26].

### 2.4. Construction of the Protein-Protein Interaction (PPI) Network

To explore the protein and protein interactions among the key targets and illustrate the underlying mechanism, the PPI network was performed and visualized utilizing the Cytoscape software and Metascape online serve, which contains six PPI online serve sourceSTRING (https://string-db.org/) and Metascape online database servers were performed to obtain the associated analysis results of predicted protein interactions [27].

The method of central network evaluation is prevalently acknowledged as the most common and master measure for screening core proteins in PPI networks. Initially, the PPI networks of BXD targets and CAG-associated targets were integrated into an intersection as key targets. Subsequently, the Cytoscape plugin, STRING, and Metascape were conducted for assessing the intersection.

### 2.5. Validation of the Binding Capacity Between Active Ingredients and Key Targets by Molecular Docking

Computer-aided drug design, development, and target prediction have recently emerged as an important method for understanding biological regulatory mechanisms, which provides a theoretical basis for the design and discovery of new drug targets. AutoDock 1.5.6 (http://autodock.scripps.edu/) and instadock (https://hassanlab.org/instadock) are gratuitous and brilliant software for drug discovery with excellent docking accuracy and speed that combines predictive physics-based methods with machine learning techniques to accelerate drug discover [27–29]. The structures of active ingredients obtained from PubChem (https://pubchem.ncbi.nlm.nih.gov/) were prepared and optimized using ChemOffice and OpenBabel software for structure optimization, format conversion, charge correction, and energy minimization [30]. The PDB files of enzymes from tryptophan metabolism with the best structural resolution coupled with endogenous ligands were downloaded from the RCSB Protein Data Bank (https://www.rcsb.org/) and were predicted using the AlphaFold database, which is a state-of-the-art AI system developed by DeepMind that computationally predicts protein structures with unprecedented accuracy and speed (https://alphafold.ebi.ac.uk/) [31]. The flies with PDB formats of key targets were subsequently optimized by Discovery Studio 4.5 to perform hydrogenation and structural modification procedure. The parameters for the grid box and docking pocket were collected from the published report, and PyMOL 2.2.0 was used to obtain boxes from the selection plugin to obtain grid box parameters. After setting the grid parameters for the protein binding pocket, a genetic algorithm was implemented, and docking run options were set to the default parameters; eventually, the dpf file was exported. The docking results were visualized utilizing Discovery Studio Visualizer 4.5 for docking pattern visualization.

### 2.6. Molecular Dynamics (MD) Simulation

In the validation of the Binding Capacity Between Active Ingredients and Key Targets by Molecular Docking Simulation parameters, during the protein-ligand complex simulation, all proteins were utilized amber99sb-ildn force field to process protein, and small molecules were processed with acpype (http://bio2byte.be/acpype) to generate gro and itp files [32].

After the docking procedure for obtaining optimal conformation, the molecular dynamics (MD) simulations were conducted utilizing GROMACS 2020.6 software; TIP3P was selected as the force field of water molecules. The simulation box was set at 1.0 nm to ensure the distance between the atoms of the protein-ligand complex, and the edge of the box is appropriate for periodicity conditions. Fill the entire box with water using the solvate command, and add SOL items to the molecules section of the top file after running and add ions, default add NA and CL; -neutral command was performed to balance the simulation system to neutral. Then, the steepest descent method was performed to simulate and optimize the system for energy reduction; subsequently, the energy minimization and duration 10 ns constraint dynamics was conducted. Eventually, the index file was created, and md simulation was performed for 200 ns. All MD simulations were performed under an isothermal and isostatic ensemble with a temperature of 298.15 K and a pressure of 1 atmosphere. The temperature and pressure were controlled by the V-rescale and Parrinello-Rahman methods, respectively, and the temperature and pressure coupling constants were 0.1 and 0.5 ps, respectively. Except for the protein prodrug ligand simulation time of 50 ns, the MD simulation time of the other three systems was 200 ns.

It can be applied to each compound.

### 2.7. Binding Free Energy Calculations using the Born Surface Area (MM/GBSA) Method

Eventually, the MMPBSA process in GROMACS was utilized to calculate the binding energy, and the following equation was utilized: ΔGbind = Gcomplex − Gfree‐protein − Gfree‐ligand.

MM is van der Waals and electrostatic energy (ΔGvdw + ΔGele); PB is polar solvation (ΔGpolar); SA is nonpolar solvation (ΔGnonpolar).

In the MM/GBSA calculations, the protein-ligand binding free energy is calculated based on MD simulation trajectories and compared with experimental binding data to build and validate the new model. The free energy changes during ligand-protein binding to form complexes are described by the original MM/GBSA according to the equations as the sum of different interactions. The basic principle is to calculate the difference between the bound and unbound free energies of two solventized molecules or to compare the free energies of different solventized conformations of the same molecule.

## 3. Results

### 3.1. Target Prediction and Functional Analysis of the Regulatory Effects of BXD on CAG

To collect and screen potentially druggable compounds from BXD, TCMSP online databases (https://tcmspw.com/index.php) were utilized for online searching. Based on the four predicted parameters of drugs including oral bioavailability (OB), drug-likeness (DL), toxicity prediction, and Caco-2 parameters obtained through ADME, ninety-two ingredients were selected as potential druggable active compounds of BXD, and the detailed information and structures were presented at (). Subsequently, the Venn diagram of ingredients was conducted. We found that there are a total of 182 potential active druggable ingredients in BXD, 15 ingredients in Banxia, 22 ingredients in Renshen, 5 ingredients in Shengjiang, 92 ingredients in Gancao, 14 ingredients in Huanglian and 36 ingredients in Huangqin which were identified out. The composition and content ratio of druggable potential in BXD were confirmed by a previous study which performed an LC-MS analysis to identify the principal characteristic peaks associated with a BXD fingerprint. Saponins, flavonoids and alkaloids were identified as the master abundant compounds that mainly exist in Renshen, Gamcao, Huangqin, and Huanglian, which is consistent with our results (Figures 1(a) and 1(b)) [33, 34].

### 3.2. Network Construction and Enrichment Analysis of Key Targets

After collecting the CAG-associated targets from six sources, the disease targets were taken at the intersection with BXD predicted targets to obtain key targets of BXD on CAG. There are a total of 134 key targets screened out, and the detailed target information is presented in Figure 2(a).

To explore the potential mechanism of clinical therapeutic effects of BXD on CAG, GO-related biological processes, cellular components, molecular functions, and KEGG pathways enriched analysis were performed on Metascape online serve by importing 134 key targets and, respectively, submitting enrichment analysis. To obtain better visualization of enrichment analysis, Rstudio was utilized to present Go and KEGG enrichment results (Shown in Figures 2(b)–2(d)). The enrichment analysis results indicated that the key targets were mainly enriched into 10 biological processes including cellular response to chemical stress, response to oxidative stress, and cellular response to oxidative stress biological process. The molecular function was mainly involved in protein serine/threonine kinase activity, phosphatase binding, and endopeptidase activity. The cellular component results suggested that these 134 key targets were dominating existing in membrane raft, membrane microdomain and membrane region. Moreover, the KEGG pathways (Figure 3) were enriched into TNF signaling pathway, cellular apoptosis, PI3K-Akt signaling pathway, C-type lectin receptor signaling pathway, and NF-kappa B signaling pathway, which were involved in Gastric mucosa inflammatory response, cellular apoptosis, and integrity of gastric mucosa cells, exerting a crucial role in CAG disease.

### 3.3. Analyses of the Key Target-Based Specific Protein Interaction Network

To explore the protein interaction of 134 key targets that BXD involved in the treatment of CAG, the gene list of targets was imported on Metascape and String online serve (Figure 4(a)). The protein and protein interaction (PPI) result demonstrated that the key targets were clustered as Figure 4(b) and the master protein clusters were involved in pathways in cancer, gastrin signaling pathway, and MAPK signaling pathway. These pieces of evidence revealed that BXD may exert a therapeutic role on CAG by regulating the protein interactions of the gastrin signaling pathway and MAPK signaling pathway.

### 3.4. Molecular Docking of Ingredients and Targets

To probe into the potential mechanism of BXD on CAG, the small molecules that filtered with the properties of drug properties were screened out for performing molecular docking procedures with key targets in CAG. All the pdb formats of targets were collected from RCSB Protein Data Bank (https://www.rcsb.org/), and the parameters of binding pocket of targets were obtained from the PyMOL 2.2.0 software. Eventually, the molecular docking procedure was performed by utilizing Vina software. The hot map (Figure 5) demonstrated that three targets encompassing NR3C1, NOS2, and IL-2 displayed impressive binding energy with the compounds from BXD, and it is worth noting that these compounds who represent considerable binding energy with the inflammatory targets were majorly originated from Huanglian, Huangqin, and Gancao, which was consistent with previous studies. Subsequently, we selected three target-ligand complexes to visualize the binding pattern, and the results were present. The visualization of three target-compound complexes was presented and analyzed by the Discovery studio 4.0 visualizer, and the binding pattern of NR3C1-coptisine indicated that there are three binding interactions encompassing van der vaals, Pi-Alkyl, and Pi-Pi T-shaped, which constituted the hydrophobic pocket contributing to the relatively low binding energy. In the dissection of the binding pattern of NOS2-palmidin A, three hydrogen bonds were observed interacting with TRP372, MET374, and SER242. These amino acid residues of NOS2 constitute a hydrophilic pocket that strongly interacts with the hydroxyl group of palmidin A. In the dissection of the binding pattern predicted in Discovery Studio presented in the 3D and 2D graphs, 2 hydrogen bonds between IL-2 and licocoumarone were observed. In the complex of IL-2 and licocoumarone, CYS31 (2.95 Å) and GLN74 (3.27 Å) interact with the hydroxide radical group of licocoumarone, forming 2 hydrogen bonds; moreover, PHE78 and LEU70 constitute the hydrophobic pocket that is beneficial to the stabilization of the complex (Figures 6(a)–6(f)). Based on the results described above, the conclusion could be drawn that coptisine, palmidin A, and licocoumarone could constitute stable complexes with NR3C1, NOS2, and IL-2 with low binding free energy and good binding pattern, which subsequently explored and unveiled the potential compound-target pharmacological interaction.

### 3.5. Molecular Dynamics Simulations and Analysis of Molecular Dynamics Trajectories

Subsequently, Gromacs-2019.5 was used to perform protein-ligand complex molecular dynamics simulation (MDS), which is beneficial for evaluating the stability of the ligand and protein complex. Based on the docking scores between 152 druggable compounds from BXD and selected key targets coupled with the visualization of binding pattern, three complexes including NR3C1-coptisine, NOS2-palmidin A, and IL-2-licocoumarone were selected, and their conformational behaviour was analyzed via molecular dynamics simulations and MMPBSA calculations (displayed in Figures 7(a)–7(i)). During the 100 ns molecular dynamics simulation, coptisine, palmidin A, and licocoumarone exhibited a wide range of interactions with various residues at the binding site, suggesting that three ligands form a stable complex with NR3C1, NOS2, and IL-2. Additionally, the root-mean-square deviation (RMSD) of the protein backbone and coptisine, palmidin A, and licocoumarone was of low magnitude, ranging in fluctuation, which is another strong indication of conformational stability that the protein had achieved with the ligand molecules. After analyzing hydrogen bond formation in the 100 ns of MDS, coptisine, palmidin A, and licocoumarone form 1, 2, and 2 hydrogen bonds with NR3C1, NOS2, and IL-2, respectively, as indicated by the docking pattern. Subsequently, we utilized molecular mechanics Poisson Boltzmann surface area calculations (MMPBSA) to obtain the van der Waals energy, electrostatic energy, polar solvation energy and SASA energy of coptisine, palmidin A, and licocoumarone complexed with NR3C1, NOS2, and IL-2, where positive values are unfavorable for interaction and negative values are favorable. In the MMPBSA calculations, the total binding free energy of -63.180, -52.778, and -43.012 kcal/mol, suggesting the strong interactions between protein ligands and high stability of the complexes formed.

### 3.6. Free Energy of Binding and Interacting Residue Results in Molecular Dynamics Simulation

Binding free energy is of great importance in the drug discovery process which could provide more accurate and detailed energy information [35]. A host of methods for calculating the binding free energy has been put forward in the last decades, for example, Thermodynamics Integration (TI), Free Energy Perturbation (FEP, MM/PB(GB)SA), and Linear Interaction Energy (LIE). The method of MM/PB(GB)SA is widely acknowledged as the most common and prevalent approach for calculating receptor-ligand binding free energy by researchers [36]. The main principle of program calculation of molecular Mechanics/Poisson Boltzmann (Generalized Born) Surface Area is to split the binding free energy into a molecular mechanics term and solvation energy. The underlying mechanism is to evaluate the discrepancy between the binding free energy of two solventized molecules in bound and unbound states, as well as to calculate the free energy of the same molecule in different solvated confirmations. After conducting the molecular dynamics simulation procedure, the md trajectories were utilized for the free energy of binding calculation, and the results of the contribution of amino acid residues to the ligand-protein binding energy are shown in (Figures 8(a)–8(c)).

## 4. Discussion

TCM has unique therapeutic efficacy in clinical practice; many traditional Chinese prescriptions have been utilized to treat CAG, encompassing Zuojin Pill, Moluodan, and BXD [9, 37, 38]. Particularly, BXD has been widely utilized for treating various treatments of gastrointestinal diseases, including delayed diarrhea, ulcerative colitis, and ethanol-induced chronic gastritis, and exerted prominent therapeutic effects [11, 39]. Increasing emerging evidence has confirmed the anti-inflammatory and antitumor effects of the natural ingredients in BXD; additionally, the master compounds including baicalin and berberine have been identified and validated the treatments on CAG by various LC-MS analyses and pharmacological research. Nevertheless, in comparison with the precise clinical efficacy and the long history of the application of TCM, there is a relative lack of research on the mechanism of TCM. Accordingly, considering the multicomponent and multitarget characterization of TCM, the method of network pharmacology has been applied to study the potential mechanism of TCM and a series of progress was accomplished [40, 41]. In our current study, we initially explored the potential mechanism of BXD on CAG via the method of network pharmacology considering the definitive clinical efficacy of BXD.

TNF signaling pathway, PI3K-Akt signaling pathway, and NF-kappa B signaling pathway are common inflammatory associated pathways that CAG is involved in, and many traditional Chinese medicines have been reported to modulate these inflammatory pathways. For example, NF-kappa B and TNF signaling pathway have been reported to be associated with the helicobacter pylori gastrointestinal infection in CAG, and many traditional Chinese medicines have accomplished good results in the anti-inflammatory treatment of gastritis which encompassing Gancao, Huanglian and Huangqin [42–47]. Additionally, various herbal natural compounds have been reported for their anti-inflammatory pharmacological effects in the treatment of gastritis and have been developed as clinical agents, for example, 18*β*-glycyrrhetinic acid (GRA) demonstrated in vivo pharmacological effects in the treatment of H. pylori gastritis infection. Berberine and baicalin also have been demonstrated in the treatment of CAG [48–50]. Consistently, the network pharmacology results from our study suggested that there are a total of 152 druggable ingredients in BXD and the target enrichment analysis demonstrated that the major pathways BXD involved in treating CAG were TNF signaling pathway, cellular apoptosis, PI3K-Akt signaling pathway, C-type lectin receptor signaling pathway, and NF-kappa B signaling pathways. These pathways are closely associated with the inflammatory response and the gastrointestinal environment.

The interactions of proteins are of crucial importance in normal biological processes. Cells receive signals from exogenous or endogenous sources and regulate their gene expression through their specific signaling pathways in order to maintain their normal biological properties. Proteins play an important role in this process, as they can internally regulate and mediate many biological activities of the cell. Although some proteins can function as monomers, most proteins act with chaperone molecules or form complexes with other proteins to perform their functions [51]. Accordingly, the protein interaction results also suggested the therapeutic role of CAG by regulating the protein interactions of the gastrin signaling pathway and MAPK signaling pathway. Considering that most small-molecule drugs exert their therapeutic effects mainly by acting on receptors to activate or inhibit. Remarkably, interactions between drugs and targets are the basis of biological effects. Many interaction modes exert a crucial role in the identification and binding of proteins and drugs [52]. However, they differ in stability and binding due to differences in binding energy and effective radius. In this study, three master interaction modes are introduced as described previously. Hydrogen bonding, with an average binding energy of 5 kJ/mol, is a weak electrostatic attraction between an electronegative hydrogen atom and an electronegative heteroatom and plays an important role in drug-target interactions. With the development of structural biology and computational chemistry, more and more natural compounds are being revealed for their pharmacological effects and developed as small molecule drugs, which accelerated drug development and mechanism discovery. Therefore, we attempted to explore the therapeutic effects of BXD on CAG from the perspective of drug-target interactions via the method of molecular docking and molecular dynamics simulation. After the docking procedure between 152 ingredients and selected key targets, the compounds with better results in docking with inflammatory targets were mostly from Gancao, Huanglian, and Huangqin herbs in BXD. Subsequently, molecular dynamics simulation was performed to validate the activity and stability of the active ingredient and the target protein during the binding process and calculate the contribution of amino acid residues to the binding free energy. The results demonstrated that palmidin A, licocoumarone, and coptisine could form stable complexes with NOS2, IL-2, and NR3C1, providing a theoretical basis for drug development and mechanism study of BXD for CAG.

There are some limitations in our study. First, we did not perform the relevant assays to determine the effect of BXD on CAG. Besides, the relation of BXD and signaling pathways and protein complexes was not verified by experiments. All these limitations will be perfected in the future study.

In conclusion, our study elucidated the potential mechanisms of BXD underlying CAG via network pharmacology, molecular docking, and molecular dynamics simulations, which might provide theoretical value for the treatment of CAG.

## Figures and Tables

**Figure 1:** (a) The Venny plot of druggable ingredients from six herbs of BXD. (b) The UpSet graph coupled with elements of ingredients from six herbs of BXD.

**Figure 2:** Go and KEGG pathways analysis. (a) Intersection diagram of BXD predicted targets and CAG-related targets. (b–d) GO-related biological processes, cellular components, and molecular functions enrichment analysis of key targets.

**Figure 3:** The KEGG pathway enrichment analysis of key targets. The squares represent target and pathway information, respectively, and the pathways are sequenced by gene ratio.

**Figure 4:** Graph of protein-protein interactions. (a) General view of the interactions of proteins and clustered proteins. (b) Five protein clusters are associated with the Gastrin signaling pathway, MAPK signaling pathway, Apoptosis, G alpha (q) signalling events and collagen catabolic process. These circles represent the target protein, and the line represents the interaction of the target protein.

**Figure 5:** Heat map of docking energies.

**Figure 6:** The interaction profile for three complexes. (a–c) Overall structure of NR3C1-coptisine, NOS2-palmidin A and IL-2-licocoumarone complex, (2d) binding modes of NR3C1-coptisine, NOS2-palmidin A, and IL-2-licocoumarone were presented as (d–f).

**Figure 7:** The RMSD results and Hbonds analysis of NOS2-palmidin A, NR3C1-coptisine, and IL-2-licocoumarone complex. (a–c) The RMSD of NOS2, RMSD of palmidin A relative to NOS2, and change in the number of hydrogen bonds during 100 ns simulation. (b–d) The RMSD of NR3C1, RMSD of coptisine relative to NR3C1, and change in the number of hydrogen bonds during 100 ns simulation. (d–e) The RMSD of IL-2, RMSD of licocoumarone relative to IL2, and change in the number of hydrogen bonds during 100 ns simulation.

**Figure 8:** The graph of free energy contribution of amino acid residues to ligand-protein binding in three protein-ligand complexes.

## Data Availability

Data appear in the submitted article.
